# Perioperative Fast-Track Surgery Nursing Intervention for Patients with Kidney Stone Disease under Computed Tomography Imaging

**DOI:** 10.1155/2023/1101388

**Published:** 2023-02-06

**Authors:** Yingmei Chen, Jun Yang

**Affiliations:** Department of Urology Surgery, Honghu Traditional Chinese Medicine Hospital, Honghu, Jingzhou 433200, Hubei, China

## Abstract

This research aims to analyze the clinical intervention effect of perioperative fast-track surgery (FTS) nursing on patients with kidney stone disease (KSD) under computed tomography (CT) imaging. One-hundred KSD patients were selected as research objects and grouped after CT examination. These objects were randomly divided into a research group (FTS nursing intervention, *n* = 50) and a control group (general routine nursing intervention, *n* = 50). The preoperative psychological status of patients was compared between the two groups, using Self-rating Anxiety Scale and Self-rating Depression Scale. The hunger and thirst situations were compared using Numerical Rating Scale; postoperative recovery time, incidence of complications, and nursing satisfaction were also compared. The high-density shadow could be clearly observed in the right kidney of the patients in the CT imaging examination. The nursing outcomes suggested that there was no notable difference in hunger between the two groups, and anxiety, depression, and thirst in the research group were highly better than those in the control group (*P* < 0.01). The time of the first exhaust, the time of body temperature returning to normal, the time of getting out of bed, and the length of hospital stay in the research group were all shorter than those in the control group (*P* < 0.05). The total postoperative satisfaction of the research group (98.00%) was greatly better than the 88.00% in the control group (*P* < 0.05). As the FTS concept was applied in the perioperative nursing of KSD patients under CT imaging, the preoperative and postoperative negative emotions of patients could be improved. Thereby, the postoperative recovery rate of patients was promoted, postoperative complications and patients' pain were reduced, and the postoperative quality of life of patients was also improved.

## 1. Introduction

Kidney stone disease (KSD), also called renal calculus and nephrolithiasis, is caused by the abnormal accumulation of the precipitated crystals in the kidneys [1]. It occurs when the increase in the concentration of crystal substances (such as oxalic acid and uric acid) or the decrease in the solubility of the substances in the urine exceeds the saturation level. Today, the most common disease in clinical urology is lithiasis in the urinary system, of which KSD accounts for 80%. KSD is more common in men, and more than half of the patients are prone to recurrence after 5 years. Some patients often manifest with nausea, vomiting, hematuria, and other obvious clinical symptoms, and a small number of patients have no obvious clinical symptoms [2]. Patients with KSD are prone to complications such as urinary tract infection and ureteral obstruction, which seriously damage the renal function and affect the quality of life of patients. Therefore, KSD patients need to be detected, diagnosed, and treated as early as possible to avoid the physical harm caused by continuous development of the disease [3, 4]. Currently, computed tomography (CT) examination is the preferred imaging examination for the diagnosis of KSD. It is easy to operate, has no incision, and is safe. It can help the attending doctor to find the location and size of the stones accurately and allows clear observation of the morphological features of the stones. Thus, CT can provide a reliable pathological basis for the clinical diagnosis of KSD [5, 6].

With the development of science and technology, minimally invasive techniques in urology have also developed rapidly. More than 90% of KSD can be treated by minimally invasive surgery, among which percutaneous nephrolithotomy (PCNL) is the most effective minimally invasive procedure for larger stones and complex stones [7, 8]. However, PCNL may still result in multiple complications, such as intraoperative and postoperative major bleeding. The incidence of nephrectomy due to surgical major bleeding can reach 3.5%, the incidence of liver and pleura injuries is 4.3%, and that of intestinal injury is 7.8% [9, 10]. The incidence of complications due to PCNL reaches 37% worldwide. The learning process of PCNL is long, and the selection and establishment of renal puncture route determine the risks of surgery and the stone clearance rate [11]. The surgical procedure of PCNL is simple, safe, and effective but its requirements for perioperative nursing are still very high [12]. The concept of fast-track surgery (FTS) was researched and proposed by Danish doctor Kehlet in the 1990s, aiming to improve the existing preoperative and postoperative medical nursing under the premise of patients' safety. The nursing measures that are beneficial to the patients' physical and psychological health and to speeding up of recovery are adopted. FTS combines multiple disciplines such as surgery, nutrition, and rehabilitation therapy, which not only ensure patients' safety but also effectively reduce intraoperative and postoperative pain stress and complications [13, 14]. Through rigorous selection of patients, preoperative psychological counseling and education, prevention of excessive medication, comprehensive pain nursing, moderate exercise after surgery, recovery of diet in a short period, and other methods can be taken for the nursing for patients. Therefore, postoperative pain and various stresses in patients can be reduced or avoided, and the recovery of patients can be speeded up in a more effective and reasonable way [15].

Any invasive surgery has certain risks. Although PCNL is simple to operate, appropriate and effective nursing measures should be selected in the perioperative period, to reduce the postoperative complications, improve the prognosis, and speed up the recovery process of patients [16]. Therefore, on the basis of the diagnostic results of CT imaging, FTS nursing intervention was performed for patients with KSD surgery during the perioperative period. The clinical application value of FTS nursing for KSD patients in the perioperative period was determined by analyzing the relevant indicators such as the incidence of complications and postoperative recovery.

## 2. Materials and Methods

### 2.1. General Information

One-hundred KSD patients who were admitted to hospital from January 2021 to January 2022 were selected and randomly divided into research group (FTS nursing intervention, *n* = 50) and control group (general nursing intervention, *n* = 50). There was no significant difference in their general data (age, gender, lesion location, education level, etc.) between the two groups (*P* > 0.05). Therefore, there was a comparability in the research. This study was approved by ethics committee of hospital. The patients and their families signed the corresponding informed consent forms.

Inclusion criteria required the patients to have clinical manifestations of KSD and need PCNL with a holmium laser. The patients should have neither blood system diseases nor infectious diseases.

Exclusion criteria were listed as follows: those did not meet the indications for the surgery, those were complicated with malignant tumors or hematological diseases, those were accompanied with severe disturbance of consciousness, and those were women who were pregnant or breastfeeding.

### 2.2. General Flowchart

The overall flowchart of this research is shown in Figure 1.

### 2.3. CT Examination

All the patients underwent CT examination. The dual CT scanner was used for examination. The patient was in a supine position. Scanning parameters were composed of voltage 120 kV, current 130 mA, slice thickness 7 mm, and interslice distance 10 mm. For enhanced scan, contrast agent Ultravist was intravenously injected, with the specification of 300 mgI/mL, the dose of 1.5–2.0 mL/kg, and the injection rate of 1.5–2.0 mL/s. The scanning mode was the whole abdominal scan, and delayed sweep was made after 0.5 hr.

The following general requirements were stated for CT examination in patients with KSD. First, according to the patients' renal condition, the time of urography scan was decided by the radiologist. For patients with no hydronephrosis, it could be appropriately delayed for 15–30 min; for patients who have hydronephrosis, generally, a delay of 1–3 hr was allowed with the upper limit of 6 hr. Second, before the formal examination, the patients should keep an empty stomach, drink water appropriately, and exercise more. Drinking water could dilute the urine and prevent it from crystallizing. Third, the patients could be instructed to hold back the urine properly, so that the bladder was in a full state. When the bladder was in a moderately full state, both kidneys were scanned using a CT machine, and it was observed whether the patient had renal stones with the CT images. Fourth, it should be noted that gastrointestinal angiography should not be performed within 1 week before CT examination in patients with KSD. This was to avoid the interference of barium sulfate chemical reagents on surrounding normal tissues and organs, which might affect the results of kidney stone examination.

### 2.4. Nursing Methods

The routine nursing was given in the control group. Before surgery, the medical staff should inform the patients and their families about the surgical process and related precautions in detail. The medical staff arranged the patients to complete various preoperative examinations, to ensure that the physical condition of patients was tolerant to the surgery and the patients had the conditions to receive the surgery. The medical staff also assisted patients with all preoperative preparations. The attending doctor should also instruct the patients to fast for 12 hr with no drinking 4 hr before the surgery. The gastrointestinal preparation was well made, and an enema was performed if necessary. After surgery, the attending doctor should routinely and rationally use antibiotics to prevent infection and gave patients corresponding diet, exercise, and other instructions. The nursing staff should follow the doctor's instructions. In the meanwhile, the ward should be ventilated regularly, disinfected, and sterilized regularly everyday, the room temperature should be controlled, and a sterile resting environment should be provided for patients.

The FST nursing was conducted in the research group. First, for the preoperative nursing, mental nursing was carried out for patients during the entire perioperative period before, during, and after surgery, and the patients' psychological status should be always concerned. For functional exercise and nutritional support, patients were encouraged to perform activities such as climbing stairs as early as possible under the guidance and help of medical staff. Parenteral or enteral nutritional support was given in combination with the patients' own physical condition, to increase the resistance of patients and lay a good foundation for postoperative recovery [17]. For dietary nursing, medical staff should instruct patients to drink water and carbohydrates 2 hr before surgery to improve preoperative discomfort symptoms.

Second, intraoperative nursing consisted of anesthesia nursing and body temperature preservation nursing. For anesthesia nursing, anesthesia personnel should choose an appropriate anesthesia method depending on the patients' own situation. Short-acting anesthetic drugs should be applied as possible to achieve the quick onset and quick recovery. After anesthesia, the medical staff adjusted the patients' position to a suitable state for the surgery. During the PCNL surgery, the assistant nurse should strictly observe the patients' heart rate, blood pressure, and other vital signs, and immediately inform the surgeon if there was any abnormality [18]. For body temperature preservation nursing, the temperature and humidity of the operating room were adjusted to the optimal in advance. The infusion and cleaning solution was placed in an incubator in advance for warming. It should be noticed to keep the patients' limbs warm and avoid the stress response due to hypothermia.

Third, postoperative nursing included drainage nursing, puncture point nursing, pain nursing, and early activity and eating. For drainage nursing, the daily drainage volume, and the nature and color of the drainage fluid were closely observed and recorded. If the drainage fluid was bright red, the nursing staff should inform the doctor in charge immediately. Antibiotics were given for routine anti-infection as prescribed by the doctor, to avoid postoperative complicated infection. For puncture point nursing, it was closely observed whether the puncture point was exuding fluid, blood, or leakage after surgery. If the above situations occurred, the puncture point should be disinfected and the dressing should be replaced in time to avoid infection of the puncture point [19]. For pain nursing, the postoperative pain degree of patients was evaluated according to their facial expression, language, etc. It was decided to give analgesic drug treatment depending on the patients' pain degree. For early activity and eating, patients were encouraged to get out of bed early and perform functional exercises during the recovery period from surgery to prevent the deep vein thrombosis [20]. After patients were able to eat, they should eat more cellulose-rich and easily digestible foods, to reduce the burden on the gastrointestinal tract, promote gastrointestinal motility, and speed up food digestion.

### 2.5. Observation Indicators

Preoperative discomfort was compared between the two groups, including the depression, anxiety, hunger, and thirst. The degrees of anxiety and depression were evaluated using the Self-rating Anxiety Scale (SAS) and the Self-rating Depression Scale (SDS).

Postoperative recovery time was compared between the two groups. The indicators were composed of the time of the first exhaust, the time of body temperature returning to normal, the time of getting out of bed, and the length of hospital stay.

A comparison of complications was also made between the two groups. The complications were bleeding, abdominal distension, infection, urinary extravasation, deep vein thrombosis, etc.

The nursing satisfaction was compared between the two groups (generally satisfied was included in satisfied). The calculation method of nursing satisfaction is given in Equation (1):

(1) $$\begin{array}{c} \text{Nursing satisfaction}=\frac{n_{1}+n_{2}}{N}, \end{array}$$

where *N* represents the total number of patients, *n*_1_ represents the number of satisfied patients, and *n*_2_ represents the number of generally satisfied patients.

### 2.6. Statistical Analysis

SPSS 22.0 was applied for analyzing the data in this research. The measurement data (time to first exhaust, time to return to normal body temperature, time to get out of bed, and length of hospital stay) were tested using Shapiro–Wilk normality test and Bartlett's homogeneity test for variance. All the measurement data were confirmed to have homogeneity of variance and obeyed approximate normal distribution, then expressed as mean ± standard deviation ($\bar{x}\pm s$) as *t*-test was utilized. The enumeration data (the incidence of complication and nursing satisfaction) were expressed as rate (%), *χ*^2^ test was adopted, and the test level was *α* = 0.05.

## 3. Results

### 3.1. CT Imaging Diagnosis Results

The CT examination outcomes of patients with KSD is shown in Figure 2. Figures 2(a) and 2(b) were horizontal images, while Figures 2(c) and 2(d) were coronal images. There was a high-density shadow in the right kidney of the patient, bilateral ureters and bladder were not abnormal. Thus, this high-density shadow was a kidney stone.

### 3.2. Comparison of Preoperative Discomforts

One-hundred patients with KSD were randomly divided into the research group (*n* = 50) and the control group (*n* = 50). The discomforts of two groups of patients before surgery were compared. There was no difference in hunger between the two groups, while the anxiety, depression, and thirst in the research group were significantly better than those in the control group (Table 1).

### 3.3. Comparison of Postoperative Recovery Time

The postoperative recovery time was compared between the two groups. The time of first exhaust, the time of body temperature returning to normal, the time of getting out of bed, and the length of hospital stay in the research group were all shorter than those in the control group (*P* < 0.05) (more details are shown in Table 2).

### 3.4. Comparison of Complications

The postoperative complications, occurred in patients, were compared between the two groups. The conditions of bleeding, abdominal distension, infection, urinary extravasation, and deep vein thrombosis in the research group were markedly better than those in the control group. The total incidence of complications was 8.00% in the research group, much lower than that in the control group (24.00%), which is shown in Table 3.

### 3.5. Nursing Satisfaction of Patients

The satisfaction of patients after nursing was compared between the two groups. The total satisfaction of the research group was 98.00%, which was remarkably higher than 88.00% of the control group (Table 4).

## 4. Discussion

As a common disease in urology, KSD has a high morbidity and poor prognosis, which seriously affects the normal life and work of patients. To increase the diagnosis rate of KSD and treat it as soon as possible, researchers have developed an accurate, scientific, and rapid diagnostic measure. It is of great significance to improve the curative effect and the prognosis of patients [21]. In the past, due to the limitation of science and technology, abdominal plain film, X-ray, intravenous urography, and other methods were mostly used for the diagnosis of KSD. In recent years, with the rapid development of imaging technology in China and the continuous research of KSD, the spiral CT technology and three-dimensional reconstruction software have been greatly improved. The multislice spiral CT, with outstanding achievements, has gained more and more clinical applications because of its advantages of short time-consuming, noninvasion, and fast scanning [22]. In recent years, the application of the digital model of urinary CT three-dimensional reconstruction has gradually received attention.

Currently, surgical treatment is mainly used for KSD to remove the stones and improve the clinical symptoms of patients. However, this surgical method requires high-quality perioperative nursing. Therefore, strengthening the quality of perioperative nursing is an important guarantee for the completion of the surgery and the good prognosis of patients. The general routine nursing is mainly environmental nursing, which lacks attention to the psychological status of patients. The psychological pressure on patients is extremely high, which leads to unsatisfactory nursing effects, and patients are generally dissatisfied with the nursing effects. Gillams et al. [23] proposed the concept of FTS in 2001. This concept refers to optimizing many nursing measures during the perioperative period, so as to improve the quality of nursing, reduce the incidence of complications, shorten the length of hospital stay, and enable patients to recover quickly. Smith et al. [24] believed that fasting for 6 hr before surgery could promote postoperative recovery more than fasting for 12 hr, and water intake 2 hr before anesthesia hardly caused regurgitation and aspiration in patients. Therefore, in this research, the patients in the research group fasted for 6 hr before surgery and took 300 mL of 10% glucose orally 2 hr before surgery. Thus, not only the fasting hunger of patients was relieved but also the incidence of hypoglycemia and electrolyte imbalance was reduced. Yildirim et al. [25] thought that FTS nursing should enable patients to eat and get out of bed at an early stage, as well as restore gastrointestinal function. It should also make patients to prevent deep vein thrombosis in the lower limbs and improve oxygen content in tissues; thus, it is conducive to rapid recovery postoperatively.

As a new type of nursing, FTS nursing is more comprehensive and more humanized with more attention to the psychological needs of patients compared to routine nursing. With the improvement of patients' needs and the update of medical models, psychological issues have gradually been paid attention to in clinical practice. The preoperative psychological status can affect the surgical status of patients, which directly affect the surgical situation. Therefore, psychological intervention should be given to patients before surgery [26]. Medical staff should pay more attention to the necessity of nursing while focusing on treatment. How to further improve the postoperative effect of PCNL was the research focus, and the premise of improving the surgical effect was to improve the nursing effect.

## 5. Conclusion

FTS concept was applied in the perioperative nursing for patients with KSD under CT imaging. The application could improve the preoperative and postoperative negative emotions, raise the postoperative recovery rate, reduce postoperative complications, relieve pain, and promote the quality of life of patients after surgery. Thus, FTS was worth being promoted. However, the few research objects included and the relatively concentrated sample sources perhaps have a certain impact on the research results. Therefore, it was necessary to be improved and optimized in the follow-up research, so as to research CT imaging features and the application value of FTS nursing intervention in KSD surgery in depth.

## Figures and Tables

**Figure 1:** The overall flowchart for the research.

**Figure 2:** CT imaging results: (a) and (b) were the images in horizontal plane, while (c) and (d) were coronal images. The marked region in the figure was a kidney stone.

**Table 1:** Comparison of preoperative discomforts of patients in the two groups.

Groups	*n*	SAS score	SDS score	Hunger score	Thirst score
Research group	50	28.79 ± 1.26	28.56 ± 1.43	1.12 ± 0.65	1.28 ± 0.86
Control group	50	39.43 ± 2.15	39.45 ± 2.62	1.33 ± 0.78	3.53 ± 1.41
*t*	–	32.717	33.848	10.597	10.869
*P*	–	<0.001	<0.001	<0.001	<0.001

**Table 2:** Comparison of postoperative recovery time of patients between the two groups.

Groups	*n*	Time to first exhaust (hr)	Time to return to normal body temperature (hr)	Time to get out of bed (hr)	Length of hospital stay (days)
Research group	50	17.46 ± 3.21	3.81 ± 0.76	5.72 ± 1.12	5.35 ± 0.26
Control group	50	25.14 ± 5.32	2.19 ± 0.64	11.41 ± 1.15	7.14 ± 0.38
*t*	–	10.146	13.241	28.845	25.179
*P*	–	<0.001	<0.001	<0.001	<0.001

**Table 3:** Comparison of postoperative complications between the two groups.

Groups	*n*	Bleeding	Abdominal distension	Infection	Urinary extravasation	Deep vein thrombosis	Total incidence (%)
Research group	50	3	1	3	2	3	24
Control group	50	1	0	2	0	1	8
*χ* ^2^	–	–	–	–	–	–	4.078
*P*	–	–	–	–	–	–	0.034

**Table 4:** Comparison of nursing satisfaction of patients.

Groups	*n*	Dissatisfied	Generally satisfied	Satisfied	Total satisfaction
Research group	50	6	8	36	88
Control group	50	1	5	44	98
*χ* ^2^	–	–	–	–	4.987
*P*	–	–	–	–	0.019

## Data Availability

The data used to support the findings of this study are available from the corresponding author upon request.
